The article "Effect of Music Therapy Combined with Free Position Delivery on Labor Pain and Birth Outcomes" was retracted in 2023. Reasons: signs of a paper mill; compromised peer review; unreliable results or conclusions.

# Effect of Music Therapy Combined with Free Position Delivery on Labor Pain and Birth Outcomes

**DOI:** 10.1155/2022/8963656

**Published:** 2022-05-11

**Authors:** Huimin Guo, Mochun Que, Jie Shen, Qiaole Nie, Youguo Chen, Qin Huang, Aiying Jin

**Affiliations:** ^1^Department of Obstetrics and Gynecology, The First Affiliated Hospital of Soochow University, Jiangsu, China; ^2^Department of Physiology and Neurobiology, Medical College of Soochow University, China; ^3^Beijing Yuedi Music Analgesia Labor Institute, Beijing, China

## Abstract

**Objective:**

At present, the clinical effect of music therapy combined with free position to assist delivery is rarely reported. Based on evidence-based nursing, this study is aimed at exploring the effect of the combination of music therapy and free position delivery on labor pain and maternal and fetal outcomes.

**Methods:**

A total of 440 primiparas with vaginal delivery in the Department of Obstetrics and Gynecology of the First Affiliated Hospital of Soochow University between July 2018 and July 2019 were selected. They were divided into music therapy, free position delivery group (*n* = 201) and traditional delivery group (*n* = 239). Subsequently, the two groups were compared in terms of the Chinese Perception of Labor Pain Questionnaire (PLPQ) score, bleeding amount at 2 hours after birth, perineal injury, labor stage duration, and 1 minute Apgar score.

**Results:**

The combination group had better results of the Chinese PLPQ score, postpartum hemorrhage, and perineum condition. However, compared with traditional delivery, a longer duration of the first stage and total stage of labor was found in the combination group. Music therapy combined with free position delivery required less medical intervention during delivery, and there was no significant difference in 1 minute Apgar score between the two groups.

**Conclusions:**

Music therapy combined with free position delivery, an intervention based on evidence-based nursing, can effectively reduce maternal labor pain, postpartum hemorrhage, soft birth canal injury, and medical intervention during labor. It is, therefore, a safe intervention to assist delivery.

## 1. Introduction

Labor pain is a complex physiopsychological experience during delivery in women, and high-level and long-lasting pain will have a markedly adverse effect on delivery. It has been reported that 60% of primipara have experienced severe labor pain [1]. Unlike other types of pain, labor pain cannot be predicted and controlled and is enhanced with the progress of labor [2]. Labor pain is not only affected by physiological factors such as prostacyclin, birth canal, fetal position, and uterine contraction intensity but also involves psychological factors. To be specific, emotions such as prenatal anxiety and fear will stimulate the sympathetic-adrenal medullary system, thus leading to increased levels of pain mediators and hypoxic metabolites and ultimately increased pain intensity. Labor pain causes strong subjective discomfort of parturients. It can induce adverse birth outcomes such as maternal and fetal hypoxia and failure of a trial of labor and even maternal emotional disorders in severe cases [3]. The American College of Obstetricians and Gynecologists (ACOG) points out that after exclusion of medical contraindications, maternal needs are the sufficient indication for labor analgesia. At present, the most commonly used method of labor analgesia in clinical practice is spinal anesthesia, which takes effect quickly and blocks nerve conduction to relieve maternal pain [4]. However, it may prolong the second stage of labor and results in increased oxytocin dosage, with disadvantages such as traumatic injury, puncture risk, and anesthesia risk [5]. Therefore, it is necessary to find other safe and effective methods to assist delivery.

The article "Effect of Music Therapy Combined with Free Position Delivery on Labor Pain and Birth Outcomes" was retracted in 2023. Reasons: signs of a paper mill; compromised peer review; unreliable results or conclusions.

The World Health Organization (WHO) proposes that some relaxation skills can be used to relieve pain according to their willingness for healthy parturients who require analgesia during labor, such as progressive muscle relaxation, breathing regulation, music, meditation, appropriate exercise, and upright position [6]. Domestic and foreign scholars have reported that music can promote maternal relaxation in the early stages of labor and serve as a stimulus for uterine action in the later stages of physical exertion, reducing anxiety and pain during labor [7]. The effect of music on human physiology is achieved by stimulating the auditory center and then acting directly on the limbic system, reticular formation, hypothalamus, and cerebral cortex of the brain. Because the auditory center and pain center of the cerebral cortex are adjacent, stimulating the auditory center can inhibit the pain center, thereby reducing the level of *β*-endorphin immunoreactivity, increasing oxygen supply to tissues and organs, inhibiting the production of endogenous pain-suppressing substances and promoting the metabolism of pain-inducing substances, and ultimately decreasing pain perception [8]. Delivery in free position is recommended by WHO in *Care in normal birth: a practical guide*, and this position can reduce cesarean section, postpartum hemorrhage, and the use of painkillers and oxytocin during delivery and promote spontaneous delivery [9]. At present, the clinical effect of music therapy combined with free position to assist delivery is rarely reported, so we explored this based on evidence-based nursing.

The article "Effect of Music Therapy Combined with Free Position Delivery on Labor Pain and Birth Outcomes" was retracted in 2023. Reasons: signs of a paper mill; compromised peer review; unreliable results or conclusions.

## 2. Materials and Methods

### 2.1. Collection of Patient Information

We selected 440 primiparas who underwent vaginal delivery in the Department of Obstetrics and Gynecology of the First Affiliated Hospital of Soochow University during July 2018-July 2019. They were divided into music therapy, free position delivery (*n* = 201) and traditional delivery group (*n* = 239) according to the principle of randomized control. Inclusion criteria were as follows: (1) primipara with spontaneous vaginal delivery, (2) singleton pregnancy, and (3) no pregnancy complications. Exclusion criteria were as follows: (1) premature delivery; (2) abnormal maternal mental status; and (3) patients receiving drug analgesia, assisted vaginal delivery. Informed consent was obtained from all patients and their families, and this study was approved by the Ethics Committee of the First Affiliated Hospital of Soochow University (No. 2022-075).

### 2.2. Intervention Methods

Music therapy experts designed personalized music therapy based on maternal personal experiences and preferences. Before birth, efforts were taken to pacify the mood of primiparas. When the cervix dilated to 2 mm, the parturient patient has entered a single-room delivery room. Appropriate medical treatment such as intravenous oxytocin and artificial rupture of membranes was given during delivery based on the status of uterine contractions, progress of labor, and the requirements of family members.

In the traditional delivery group, the parturient was in a supine position during the whole stage of labor and in a semirecumbent position (50°) during the second stage of labor.

By contrast, in the music therapy, free position delivery group, in the early stage of the first stage of labor, the parturient was instructed to take the lateral decubitus position, semirecumbent position, or semi-Fowler's position, with gentle and comfortable meditation or hypnotic music for relaxation. In the middle and late stages of the first stage of labor, the parturient was instructed to choose different positions such as walking, kneeling, sitting, or lying prone on a birthing ball and change the position once in 15-20 minutes, with intense rhythmic music played. In the second and third stages of labor, lateral decubitus position or semirecumbent position (50°) was used, with parent-child music played.

The postpartum conditions of all parturients were recorded, including presence or absence of medical intervention and the length of labor.

### 2.3. Perception of Labor Pain Questionnaire (PLPQ) (Chinesized)

The perception of labor pain questionnaire [10] Chinesized and verified by Jin et al. [11] was employed for evaluating the parturient's perception of labor pain. The scale consists of 2 components (pain response and pain tolerance) including 16 items. By using Likert 5-level scoring, each item was rated as 1 (quite correct), 2 (correct), 3 (uncertain), 4 (incorrect), and 5 points (quite incorrect), respectively. The higher the score, the more severe the labor pain.

The article "Effect of Music Therapy Combined with Free Position Delivery on Labor Pain and Birth Outcomes" was retracted in 2023. Reasons: signs of a paper mill; compromised peer review; unreliable results or conclusions.

### 2.4. Apgar Score at 1 min [12]

On completion of airway clearance, amniotic fluid drying, and tactile stimulation, Apgar score was checked within 1 minute after birth. Neonates were assessed from 5 aspects: heart rate, reflex response, muscle tone, respiration, and skin color. Each item was rated as 0-2 points, with a total score of 10 points, and lower scores represent worse neonatal status.

### 2.5. Perineal Pain Score [13]

The degree of postpartum perineal tear was recorded: 0 point: third-degree perineal laceration or above, 1 point: lateral episiotomy, 2 points: median episiotomy or second-degree perineal laceration, 3 points: first-degree perineal laceration, and 4 points: intact perineum.

### 2.6. Amount of Bleeding at 2 Hours after Birth [14]

The amount of blood loss at 2 hours after birth was calculated and recorded: volume of bleeding at 2 hours after birth = blood loss in blood collection drape placed under the woman′s buttocks + (wet weight of blood − soaked dressings − dry weight of dressings)/1.05.

### 2.7. Statistical Analysis

All data were analyzed using SPSS 26.0. Measurement data were expressed as mean ± standard deviation (mean ± SD), with paired *t*-test used for comparison between the two groups. Enumeration data were expressed as frequency (*n*) or rate (%), with a chi-square test for statistical analysis. The difference was regarded as significant if *P* values < 0.05.

## 3. Results

### 3.1. General Information of Parturients in the Two Groups Had No Significant Differences

A total of 440 primiparas were included, including 201 in the music therapy, free position delivery group and 239 in the traditional delivery group. There were no significant differences in age, height, weight, gestational age, gravidity, education, occupation, and income between the two groups, indicating that the two groups were comparable (Table 1).

### 3.2. Effect of Two Delivery Modes on Maternal Labor Pain Response and Tolerance

The Chinese PLPQ score was used to evaluate the effect of the two modes of delivery on maternal labor pain. The results showed that in comparison with traditional delivery, a combination of music therapy and free position could obtain lower levels of pain response, pain tolerance, and total pain score of parturients, suggesting the combination could effectively relieve labor pain (Table 2).

The article "Effect of Music Therapy Combined with Free Position Delivery on Labor Pain and Birth Outcomes" was retracted in 2023. Reasons: signs of a paper mill; compromised peer review; unreliable results or conclusions.

### 3.3. Effect of the Two Delivery Modes on Maternal and Fetal Outcomes

The differences in the maternal and fetal outcomes between the two groups were further compared. We found the combination group had a longer duration in the first stage and total stage of labor, but the bleeding amount at 2 hours after the delivery was significantly reduced, and the perineum condition score was significantly increased. Additionally, compared with the traditional delivery, music therapy combined with free position delivery resulted in a lower proportion of parturients requiring medical intervention during delivery. But there was no significant difference in 1-minute Apgar score between the two groups of newborns (Table 3). The above results indicated that music therapy combined with free position delivery could reduce maternal labor pain and improve maternal and fetal outcomes.

## 4. Discussion

Studies of Hu [15] and Peng [16] have shown that music therapy can relieve anxiety and pain-induced stress reactions during delivery. Also, Zhang et al. [17] believe that personalized music intervention can stimulate the senses of patients through the rhythm and melody and emotions in music, thereby regulating the function of the brainstem reticular formation to achieve sedation and analgesia and improving of blood pressure and heart rate. By adopting a free position, parturients can freely change the center of gravity and adjust to a comfortable position, thus achieving the goals of relaxing the body, relieving pain and numbness in the lower back and lower limb, and diverting attention from pain to gain [18, 19]. According to our study, the humanized intervention method using music therapy combined with free position delivery could effectively reduce the perception of labor pain which was consistent with a previous study using doula combined with free position to relieve maternal delivery discomfort and anxiety [20]. Consistent results further verify that a combined therapy can successfully reduce labor pain and improve delivery experience.

From the perspective of delivery mechanism, an upright position is more helpful for fetal delivery. Because such position can maximize gravitational effects and therefore facilitate fetal descent and reduce muscle work and oxygen consumption, contributing to perineal relaxation [21] and reduction of perineal laceration. Music is a special language whose frequency, rhythm, and regular acoustic vibration produce physical energy acting on people's physiology and psychology. Music used during labor can reduce maternal excessive tension and anxiety associated with loss of confidence in delivery, excessive physical exertion, and uterine atony [22]. The uterine atony and soft birth canal injury are the two vital factors of postpartum hemorrhage [23]. The results of this study revealed that music therapy combined with free position was helpful in reducing postpartum hemorrhage and soft birth canal injury, as well as medical intervention during delivery, which is consistent with the study by Zhu [24] using music therapy to achieve decreases of duration of labor, bleeding volume, and labor pain and an increased probability of spontaneous delivery.

The article "Effect of Music Therapy Combined with Free Position Delivery on Labor Pain and Birth Outcomes" was retracted in 2023. Reasons: signs of a paper mill; compromised peer review; unreliable results or conclusions.

Some studies have reported that free position delivery can enhance the contractility of abdominal muscles, pelvic floor muscles, and limb muscle groups and thus improve uterine action. Additionally, upright position of the upper body is conducive to the fetus descent with the help of its own weight and gravity, thereby increasing head-to-cervix pressure and effective contractions and ultimately accelerating labor [25]. However, we found the combined group had a longer duration in the first stage and total stage of labor, but no significant difference was identified in the second and third stages of labor between the two groups. Our results are different from previous studies [13, 14], which may be due to the fact that compared with the traditional delivery group, the lower proportion of medical intervention with artificial rupture of membranes and intravenous infusion of oxytocin in the first stage of labor in the combined group results in labor lasting longer. This is consistent with the new standard of labor stage advocated by WHO. The new standard refers to less medical intervention during the first stage of labor, especially during the incubation period [26], and more humanistic care measures during labor such as encouraging the parturient to take a free position, stabilizing maternal mood, eating, distraction, interaction between the parturient and her family, and encouraging doula and family members to accompany patients during delivery [27]. Our findings indicate that combining music therapy with a free position delivery can successfully relieve labor pain, prevent postpartum hemorrhage, and provide a positive maternal delivery experience with no adverse effects on maternal or infant safety. Our results, however, have certain limitations, particularly in terms of the lack of systematic treatment guidelines for standardized treatment, such as music mode selection and music therapy duration. Although in terms of individualized treatment, we can provide personalized music mode for puerpera, and there is still a need to synthesize the experience and develop acceptable treatment protocols for the standardization of treatment modalities.

The article "Effect of Music Therapy Combined with Free Position Delivery on Labor Pain and Birth Outcomes" was retracted in 2023. Reasons: signs of a paper mill; compromised peer review; unreliable results or conclusions.

## 5. Conclusions

Music therapy combined with free position delivery can effectively relieve maternal mental stress and thus relieve labor pain. Such combination requires fewer medical interventions, results in less postpartum hemorrhage and better maternal delivery experience, and has no adverse effects on the safety of mothers and infants. The above results suggest that music therapy combined with free position delivery can improve maternal labor pain and birth outcomes, providing a reference for the application of this new delivery method for clinical parturients.

## Figures and Tables

**Table 1:** General information of parturients in the two groups.

Items	Music therapy, free position delivery group (*n* = 201)	Traditional delivery group (*n* = 239)	Statistics	*P* value
Age (year, x̅ss)	27.85 ± 3.53	27.99 ± 3.60	-0.401^1)^	0.688
Height (cm, x̅ss)	160.03 ± 16.59	161.76 ± 10.26	-0.790^1)^	0.404
Weight (kg, x̅ss)	58.17 ± 15.40	56.54 ± 8.02	1.420^1)^	0.156
Gestational age (week, x̅ss)	39.26 ± 0.98	39.07 ± 2.70	1.052^1)^	0.294
Gravidity (time, x̅ss)	1.36 ± 0.60	1.37 ± 0.63	-0.214^1)^	0.830
Education				
Primary school	1	0	2.648^2)^	0.754
Junior high school	6	11		
Senior high school/technical school/technical secondary school	18	17		
Junior college	78	90		
Undergraduate	82	103		
Master's degree or above	16	18		
Occupation				
Full-time wife	15	18	2.181^2)^	0.336
In-service	166	186		
Unemployed/between jobs	20	35		
Income (RMB)				
10,000 or above	21	34	3.434^2)^	0.329
5000-10,000	129	133		
2000-5000	34	50		
<2000	17	22		
Household registration				
Nonagricultural	127	137	1.474^2)^	0.225
Agricultural	74	102		

Note: 1) represents *t* value, while 2) represents *χ*^2^ value.

**Table 2:** Chinese PLPQ score of parturients in two groups.

Group	*n*	Pain response	Pain tolerance	Total pain score
Music therapy, free position delivery group	201	24.73 ± 7.28	9.93 ± 3.91	34.65 ± 10.20
Traditional delivery group	239	27.06 ± 7.49	10.40 ± 4.29	37.46 ± 10.70
*t* value		3.303	1.207	2.801
*P* value		0.01^∗∗^	0.228	0.05^∗^

Note: ^∗^*P* < 0.5; ^∗∗^*P* < 0.01.

**Table 3:** Maternal and fetal outcomes in the two groups.

Items	Music therapy, free position delivery group (*n* = 201)	Traditional delivery (*n* = 239)	*t/χ* ^2^ value	*P* value
First stage of labor (min)	478.76 ± 161.67	396.48 ± 159.21	-5.355	≤0.001^∗∗∗^
Second stage of labor (min)	60.88 ± 34.85	62.47 ± 40.92	0.441	0.660
Third stage of labor (min)	5.29 ± 3.85	6.07 ± 5.55	1.718	0.087
Total stage of labor (min)	544.93 ± 171.05	465.02 ± 170.87	-4.884	≤0.001^∗∗∗^
Bleeding amount at 2 hours after birth (ml)	234.65 ± 109.77	262.34 ± 129.27	2.430	0.016^∗^
Perineal condition score	2.50 ± 0.99	2.25 ± 1.08	-2.49	0.013^∗^
1 min Apgar score	9.89 ± 0.43	9.82 ± 0.58	1.379	0.169
Medical intervention during delivery	16 (8%)	106 (44.4%)	72.153	≤0.001^∗∗∗^

Note: ^∗^*P* < 0.05 and ^∗∗∗^*P* < 0.001 vs. traditional delivery group.

The article "Effect of Music Therapy Combined with Free Position Delivery on Labor Pain and Birth Outcomes" was retracted in 2023. Reasons: signs of a paper mill; compromised peer review; unreliable results or conclusions.

## Data Availability

The data used to support the findings of this study are available from the corresponding author upon request.
